# Evaluation of crude oil biodegradation using mixed fungal cultures

**DOI:** 10.1371/journal.pone.0256376

**Published:** 2021-08-26

**Authors:** Abeer R. M. Abd El-Aziz, Monira R. Al-Othman, Sameh M. Hisham, Shereen M. Shehata

**Affiliations:** 1 Botany and Microbiology Department, College of Science, King Saud University, Riyadh, Saudi Arabia; 2 Pharmaceutical Chemistry Department, College of Pharmacy, King Saud University, Riyadh, Saudi Arabia; Ghazi University Dera Ghazi Khan, PAKISTAN

## Abstract

The use of potent fungal mixed cultures is a promising technique for the biodegradation of crude oil. Four isolates of fungi, namely, *Alternaria alternata* (AA-1), *Aspergillus flavus* (AF-3), *Aspergillus terreus* (AT-7), and *Trichoderma harzianum* (TH-5), were isolated from date palm soil in Saudi Arabia. The mixed fungal of the four isolates have a powerful tool for biodegradation up to 73.6% of crude oil (1%, w/v) in 14 days. The fungal consortium no. 15 containing the four isolates (1:1:1:1) performed significantly better as a biodegradation agent than other consortium in a variety of environmental factors containing crude oil concentration, incubation temperature, initial pH, biodegradation time and the salinity of the medium. The fungal consortium showed better performance in the biodegradation of normal alkanes (n-alkanes) than that of the polycyclic aromatic hydrocarbons (PAHs); the biodegradation efficiency of normal alkanes of the fungal consortium (67.1%) was clearly high than that of the PAHs (56.8%).

## Introduction

Saudi Arabia is the biggest producer and exporter of oil, which involves around one-fifth of the world’s oil holds. As of late, with the advancement of the oil and shipping industry, the oil spillage and contamination from seaward oil stages, i.e., oil big tankers, offshore oil platforms have recently risen, creating a major environmental hazard in the event of spills [1]. Crude oil, important fossil fuel and non-renewable energy source. It consists of a sticky liquid where simple and complex hydrocarbons are mixed. It is a source of various types of fuels and chemical feedstock for the petrochemical industry [2]. Crude oil has recognized carcinogenic, mutagenic and teratogenic effects. It is regarded as a significant threat to ecosystems, and after a spill, it will take several years to recover from the environmental issues that result [3]. This requires the utilization of ideal strategy, such as bioremediation methods are by “environmentally friendly”, low cost, and that avoid secondary pollution in the cleaning up of crude oil spills [4]. However, in the implementation of bioremediation technology, difficulties have been experienced due to uncontrollable factors, such as the lack of active single bio-template (microorganism) always and beside the soil which a complex, dynamic and diverse environment that reflects biogeochemical cycles [5]. To overcome these limitations about bioremediation, many researchers have utilized bacterial consortia [6], and fungal consortia [7]. Fungal and bacterial consortia and mixed cultures can be promising strategies in the bioremediation of old and recalcitrant petroleum pollution [8]. Many researchers are improving fungal consortia for the complete degradation of such hydrocarbons. In these consortia, three strategies of bioremediation are represented: (1) The target hydrocarbon compound is used as a carbon source by fungi; (2) the target hydrocarbon compound is enzymatically attacked but is not used as a carbon source (cometabolism); (3) the target compound is not metabolized at all but is absorbed and accumulated within the fungi (bioaccumulation). Although fungi participate in all three strategies, they are more effective at cometabolism and bioaccumulation than at using hydrocarbons as sole carbon sources [9]. Fungi can provide powerful and unique of biodegrading action, which is very positive, based on fungal enzymes and their effecting in hydrocarbon biodegradation system. Fungal enzymes are mainly divided into two systems, namely, ligninolytic fungi or white-rot fungi (which produce lignin peroxidase (LiP), manganese peroxidase (MnP), and laccases) and non-ligninolytic fungi (which produce cytochrome P450 monooxygenase-like enzymes) [10, 11]. However, both the ligninolytic and non-ligninolytic types of enzymes, produced by *Phanerochaete chrysosporium*, participate as catalysts, with great value for developing a co-culture system with other microbes for a greater hydrocarbon biodegradation ability [12].

This study evaluated four fungal isolates which were isolated from date palm soil, individually and in various combinations to biodegrade crude oil. Additionally, the effects of a variety of environmental factors containing crude oil concentration, incubation temperature, initial pH, biodegradation time, and salinity, on the biodegradation of crude oil. Finally, we investigated the performance of the best fungal consortium on the biodegradation of normal alkanes (n-alkanes) and polycyclic aromatic hydrocarbons (PAHs) by GC–MS.

## Materials and methods

### Fungal isolates identification

Four fungal isolates were isolated from date palm soil: *Alternaria alternata* (AA-1), *Aspergillus flavus* (AF-3), *Aspergillus terreus* (AT-7), *Trichoderma harzianum* (TH-5). These isolates were identified according to the previous methodology of internal transcribed spacer (ITS) regions [13, 14].

### Crude oil biodegradation

The DCPIP (2,6-dichlorophenol indophenol) technique was utilized, with slight adjustments, for estimating the oil-degrading capacity of the fungal isolates. A conical flask inoculated by one plug (1 cm^2^) of fungal hyphae (grown for one week) was selected from a Petri dish and carried into a 250 mL conical flask with 50 mL of Bushnell–Haas broth containing Tween 80, crude oil, DCPIP (redox indicator) with volume 0.1% (v/v), 1%, 0.008 mg/50ml respectively. All of the flasks were incubated for 14 days at 30°C. After two weeks of incubation, the samples were analyzed using a spectrophotometer (Biochrom Libra S22, Victoria, Australia) at 420 nm. The same method was applied when using test tubes (triplicates). The biodegradation ability of the fungi was detected when the color of the DCPIP changed from blue to colorless [15].

### Fungal inoculum preparation

The four tested fungal isolates were cultured individually in potato dextrose broth medium (PDB) (20 g of potato and 2 g of dextrose) in 250 mL conical flasks, to which 0.1 mL of Tween-80 was added, and then incubated at 25°C for 7 days on a shaker at 100 rpm/min. There were three replicate flasks for each medium. Using a hemocytometer, the spore inoculum concentration was set to 1 x 10^6^ spore / mL, and then the fungal inoculum was ready for use. For all crude oil biodegradation tests, the fungal suspension was used as a biodegrade agent [16].

### Biodegradation of crude oil by individual fungi and fungal consortia

The crude oil (Saudi Aramco) degradation experiment was carried out using the four isolates individually and in various combinations. The combinations were divided into four groups: The first group contained individual isolate, the second group contained two isolates, the third group contained three isolates, and the fourth group contained all four isolates. The initial inoculation quantity for each group was 5 mL of fungal suspension and 45 mL mineral salt medium (MSM) [17] of each set according to the principle of equal quantities (Table 1). Initial, 45 mL of MSM in 100 mL of flasks was set with 1% crude oil. The fungal suspension (5 mL, 1 × 10^6^ spore/mL) was inoculated in the MSM. The flasks were then incubated at 30°C, 150 rpm, and 7.5 pH for 14 days, and the process was completed in compliance with [18]. The efficiency of biodegradation has been calculated [19]. All treatments, with the control, were done in triplicate.

$$\text{biodegradation}\;\text{efficiency}=\frac{\text{T}0-\text{T}14}{\text{T}0}\;\text{x}\;100$$

T0 amount of crude oil at zero time

T14 amount of crude oil after 14 days

**Table 1:** Number of consortia and groups of isolates.

Consortium No.	Groups	Inoculum volume (ml)				Name of isolate
		AF	AT	AA	TH	
Consortium 1	Individual isolate	5	0	0	0	*A*. *flavus* (AF)
Consortium 2		0	5	0	0	*A*. *terreus* (AT)
Consortium 3		0	0	5	0	*A*. *alternata* (AA)
Consortium 4		0	0	0	5	*T*. *harzianum* (TH)
Consortium 5	Two isolates	0	2.5	2.5	0	AT+AA
Consortium 6		0	2.5	0	2.5	AT+TH
Consortium 7		0	0	2.5	2.5	AA+TH
Consortium 8		2.5	0	2.5	0	AF+AA
Consortium 9		2.5	0	0	2.5	AF+AT
Consortium 10		2.5	0	0	2.5	AF+TH
Consortium 11	Three isolates	0	1.66	1.66	1.66	AT+AA+TH
Consortium 12		1.66	1.66	1.66	0	AF+AT+AA
Consortium 13		1.66	0	1.66	1.66	AF+AA+TH
Consortium 14		1.66	1.66	0	1.66	AF+AT+TH
Consortium 15	Four isolates	1.25	1.25	1.25	1.25	AF+AT+AA+TH

### Enzyme assays

At the same time, the four fungal isolates (both individually and in combinations), which were co-cultivated with crude oil as mentioned above, were also tested for enzyme activity. The enzyme level in the medium was assayed for control and treatment after 2 weeks of incubation. At 10,000 rpm and 4° C, the cultures of fungi were centrifuged and the enzyme level was determined. Cellulase activity (Cx) was determined [20]; cellulase activity (Cx) was measured as a reduction in sugar. The laccase (Lac) enzyme was estimated of the method [21] by oxidation of 2, 2-Azino-bis-3- benzthiazoline-6-sulfonic acid (ABTS). Manganese peroxidase (MnP) was estimated based on oxidation Mn^2+^ to Mn^3+^, while lignin peroxidase (LiP) was determined by the oxidation of veratryl alcohol according to [22]. Lipase activity was assayed using p-nitrophenyl palmitate (pNPP) as the substrate [23]. All enzymes assayed in this study are expressed as U/ml.

### Environmental factors

#### Influence of crude oil concentration

Five percent (2.5 ml), 10% (5 ml), 15% (7.5 ml), and 20% (10 ml) of crude oil were poured separately into 100 mL triangular flasks. Afterward, the fungal consortium (5 mL fungal suspension) was added to MSM described in section 2.4., totaling 50 ml of sample for each experiment, and the biodegradation efficiency was assessed after 7 days of fungal culture at 20°C.

#### Influence of incubation temperature

As per the optimized oil concentrations added to MSM reported in section 2.4., Incubation temperatures have been set at 15, 20, 25, and 30°C, respectively, and the biodegradation efficiency was evaluated after 7 days of fungal culture.

#### Influence of initial pH

The pH of the MSM medium was set to 6, 7, 8, and 9 with 1 mol / L of NaOH and HCl and solution, respectively. The medium included the crude oil and, the fungal consortium (5 mL) was inoculated and the biodegradation efficiency was estimated at 20°C after 7 days of fungal culture.

#### Influence of biodegradation time

The crude oil medium (MSM) was inoculated the fungal consortium (5 mL) for 5, 8, 11, and 14 days, respectively, incubate at 20°C afterward, the concentration of crude content was determined.

#### Influence of salinity

In this experiment was employed crude oil medium (ASM) [20]. The salinity was set to 15, 20, 25, 30, and 35% by adjusting the NaCl content. After that adding the fungal consortium to medium, and the biodegradation efficiency was evaluated after 7 days of fungal culture at 20°C. All of the biodegradation efficiency trials were done in triplicate with the alive fungal cultures.

#### Analysis of crude oil degradation by GC-MS

The best fungal consortium has been tested for its ability to degrade crude oil by studying its structure before and after the fungal activity. This experiment was applied, as mentioned in section 2.4. At the time of the GC-MS analysis, the sample of crude oil degradation mixed with diethyl ether at a ratio of 1:1. The samples were agitated for 1 min, and the organic layer was released to separate after 5 min. At this moment, collecting 1 mL of the supernatant (crude oil degradation) to a 1.5 mL Eppendorf tube, and centrifuged at 3000 rpm for 3 min. 1 ml of the sample was put in a glass vial. The crude oil extracted from sample was evaluated and used a flame ionization detector via a Perkin–Elmer GC Clarus 500 system (PerkinElmer: Boston, MA, U.S.). Crude oil was separated using a capillary column (30 m × 0.25 mm × 0.25 μm), with helium as the carrier gas at a fixed flow rate of 1.0 mL/min. The inlet temperature program and operating temperatures of the injector and detector were set under the conditions described in a previous study [24, 25].

## Results and discussion

### Molecular identification

After identification via morphology and microscopy properties of fungal isolates, the molecular fundamentals (ITS regions) were utilized for confirmation of fungal isolates identification by comparing with those of reference isolates in the NCBI GenBank (Table 2). The four isolates were classified as *Alternaria alternata* (AA-1), *Aspergillus flavus* (AF-3), *Aspergillus terreus* (AT-7), and *Trichoderma harzianum* (TH-5), as shown in Table 2. Based on the cluster analysis of BLAST and the ITS sequence for each fungal isolate proved that isolate AA-1 was 99% similar to *A*. *alternata* (LC164851). Using the same method, AF-3 showed 99% similarity with *A*. *flavus* (KY488467), and AT-7 showed 98% similarity with *A*. *terreus* (KJ528526), while TH-5 showed 99% similarity with *T*. *harzianum* (KC569346). The sequence of the ITS regions appeared to be a reliable molecular method for accurate fungal classification and identification [13, 26]. The ITS regions have many advantages like accurate and sensitive, lead to the identification of any kinds of fungi, such as *Aspergillus*, *Alternaria*, and *Trichoderma* at the species level [27].

**Table 2:** Identification of fungi species isolated from rhizosphere soil by sequencing of ITS1 and ITS 2 and region of 5.8S rRNA gene compared with sequences listed in the GenBank.

Fungi species of soil date palm				Fungi of gene bank		
No.	Fungi	Accession no.*	Size (bp) of ITS1-5.8S-ITS2 region	GenBank accession number	Fungi	Identity (%)
1	*Alternaria alternata*	AA-1	469	LC164851	*Alternaria alternata*	99%
2	*Aspergillus flavus*	AF-3	5842	KY488467	*Aspergillus flavus*	99%
3	*Aspergillus terreus*	AT-7	777	KJ528526	*Aspergillus terreus*	98%
4	*Trichoderma harzianum*	TH-5	591	KC569346	*Trichoderma harzianum*	99%

* Accession no. by authors.

### Crude oil biodegradation trial by DCPIP

The screening technique was dependent on the changing of color of the fungal isolates treated with the redox indicator (Table 3) although all of the fungal isolates were confirmed to possess the ability to degrade crude oil to differing levels, the best isolates were AF-3 and TH-5, followed by AT-7 and AA-1. The ability to analyze the components of crude oil compounds depends on the oxidation of a source of carbon in said components. Three markers contribute to the biodegradation phase of these fungi: The first is a changing in the color of the medium from blue to colorless; the second is the absence of crude oil in the medium; the third, in the lower part of the culture medium, produces a mass of fungal growth. Through inserting an electron acceptor such as DCPIP into the culture medium, the process of crude oil biodegradation determines the capacity of the fungi to use the substrate through analyzing the color shift of DCPIP from blue (oxidized) to colorless (reduced) [15]. There are three central keys that help recognize fungal isolates to be biodegrade agents: decolorization of DCPIP, decrease in the amount of crude oil, and the reproduction of fungi. Three fungal isolates *Aspergillus niger*, *A*. *oryzae*, and *Penicillium commune* were isolated from Saudi Arabia and Gulf of Mexico and tested by the DCPIP method. *A*. *oryzae* was the most powerful of the three isolates, according to the DCPIP method and confirmed by gas chromatography [28, 29].

**Table 3:** Biodegradability experiment (DCPIP) by test tubes and flasks.

No.	Fungal isolate	Accession no.*	Decolorization in test tubes	Decolorization in flasks
1	*Alternaria alternata*	AA-1	++	++
2	*Aspergillus flavus*	AF-3	+++	+++
3	*Aspergillus terreus*	AT-7	++	++
4	*Trichoderma harzianum*	TH-5	+++	+++

+ = Low, ++ = mild, +++ = high.

### Enzyme activity of fungal isolates and biodegradation efficiency

Analysis of variance (ANOVA) of the Cx, Lac, Lip, LIP, and MnP enzyme activities biodegradation of crude oil were reported in Tables 4–8 for 15 consortia include the individual fungi, as well as their consortia. The consortia numbers 11,12,13,14 and 15 have been highly significant for enzyme activity efficiency with *p* values less than 0.05 based on the ANOVA test. The high *T*-value of these consortia shows that both of these linear parameters have a greater effect on enzymes production. Fig 1, S1–S4 Figs obtained the normality of data could be by plotting the normal probability plot of residuals. The residual values have been described as the difference between the observed and predicted value of the regression. The experimental points associated with the proposed standard likelihood plot from Fig 1(a) indicate that the data is not distorted everywhere and complies with data normality. Plots of residuals versus fitted values were shown in Fig 1(b). The residuals are randomly distributed around the zero line, submitting there is no bias in the variance. the histogram plot with symmetric observation, moreover confirming the normality of the data Fig 1(c). The residuals are randomly scattered with monitoring order further establishing the non-bias of the data Fig 1(d).

**Fig 1:** (a) Normal probability plot for residual value, (b) residual plots against fitted value, (c) histogram of residual value, (d) residual plot against observation order of individual fungi and fungal consortium producing cellulase.

**Table 4:** ANOVA of fungal consortium producing cellulase.

Consortium No.	*T* Value	*P* Value
Consortium 1	-6.30	0.000
Consortium 2	-7.61	0.000
Consortium 3	-7.78	0.000
Consortium 4	-7.17	0.000
Consortium 5	-6.37	0.000
Consortium 6	-0.55	0.587
Consortium 7	-2.60	0.014
Consortium 8	-3.58	0.001
Consortium 9	-0.34	0.509
Consortium 10	-0.45	0.657
Consortium 11	3.22	0.003
Consortium 12	5.00	0.000
Consortium 13	11.29	0.000
Consortium 14	10.65	0.000
Consortium 15	13.37	0.000

**Table 5:** ANOVA of fungal consortium producing laccase.

Consortium No.	*T* Value	*P* Value
Consortium 1	-9.97	0.000
Consortium 2	-7.94	0.000
Consortium 3	-11.42	0.000
Consortium 4	-9.19	0.000
Consortium 5	-2.46	0.020
Consortium 6	-1.91	0.065
Consortium 7	-1.17	0.252
Consortium 8	-0.74	0.466
Consortium 9	-0.85	0.086
Consortium 10	-3.87	0.001
Consortium 11	6.78	0.000
Consortium 12	7.01	0.000
Consortium 13	9.91	0.000
Consortium 14	10.61	0.000
Consortium 15	15.54	0.000

**Table 6:** ANOVA of fungal consortium producing lignin peroxidase.

Consortium No.	*T* Value	*P* Value
Consortium 1	-1.84	0.076
Consortium 2	2.14	0.040
Consortium 3	-1.93	0.063
Consortium 4	-1.55	0.131
Consortium 5	-0.93	0.359
Consortium 6	-0.57	0.576
Consortium 7	-0.41	0.682
Consortium 8	-0.41	0.687
Consortium 9	-0.23	0.942
Consortium 10	-0.19	0.853
Consortium 11	0.84	0.406
Consortium 12	0.57	0.574
Consortium 13	1.38	0.178
Consortium 14	1.23	0.229
Consortium 15	2.25	0.032

**Table 7:** ANOVA of fungal consortium producing lipase.

Consortium No.	*T* Value	*P* Value
Consortium 1	-7.76	0.000
Consortium 2	-9.86	0.000
Consortium 3	-9.99	0.000
Consortium 4	-7.63	0.000
Consortium 5	-5.76	0.000
Consortium 6	-3.66	0.001
Consortium 7	-1.33	0.193
Consortium 8	-2.15	0.040
Consortium 9	-2.15	0.040
Consortium 10	2.15	0.040
Consortium 11	6.41	0.000
Consortium 12	7.26	0.000
Consortium 13	8.31	0.000
Consortium 14	10.35	0.000
Consortium 15	14.48	0.000

**Table 8:** ANOVA of fungal consortium producing manganese peroxidase.

Consortium No.	*T* Value	*P* Value
Consortium 1	-7.31	0.000
Consortium 2	-6.14	0.000
Consortium 3	-6.52	0.000
Consortium 4	-7.48	0.000
Consortium 5	-2.08	0.046
Consortium 6	-1.32	0.198
Consortium 7	-1.53	0.136
Consortium 8	-3.99	0.000
Consortium 9	-3.99	0.000
Consortium 10	-1.51	0.142
Consortium 11	6.64	0.000
Consortium 12	7.38	0.000
Consortium 13	8.47	0.000
Consortium 14	6.29	0.000
Consortium 15	11.50	0.000

Biodegradation mechanism depends on molecular-weight of hydrocarbon if that low can be directly absorbed because it is soluble and readily entered into microbial cells and need two steps 1) the intracellular accumulation of solubilized hydrocarbon and 2) the enzymatic degradation by fungi whereas microbial cells can digest medium-and long-chain hydrocarbon through three steps 1) production of biosurfactants and bioemulsifiers agents, 2) intracellular accumulation and 3) the enzymatic biodegradation [30]. The fungi produced multifunctional enzymes involved in the degradation of a large variety of aliphatic and aromatic hydrocarbons. In their susceptibility to fungal attack, hydrocarbon compounds vary and are usually classified in the following increasing order: polycyclic aromatic compounds > aromatic high molecular weight > cyclic alkanes > low molecular weight aromatics > branched alkanes > n-alkanes [31].

The metabolic pathways found in fungi involve substrate oxidation by cytochrome P450 (CYP) monooxygenases containing alkane -oxygenase enzymes in microsomes [32]. In general, the degradation of aliphatic and aromatic hydrocarbons occurs via the most frequently encountered mechanism of CYP monooxygenases enzymes, which are the terminal oxidases in electron transfer chains. These enzymes have been provided the electrons for the admission of one atom of oxygen inside the aliphatic chain, while the other oxygen atom is reduced to water [33]. Two of the other mechanisms are diterminal and subterminal oxidation. In the diterminal oxidation, the aliphatic hydrocarbon is oxidized into a dicarboxylic acid [34]. the molecule is oxidized into secondary alcohol as an Intermediate compound and transform ester and ketone in case of subterminal oxidation [35]. Oxidation by CYP is not the only pathway open to fungi for the biodegradation of aliphatic and aromatic hydrocarbons, considering the above mechanisms. But the recent authors demonstrated the presence of hydroxyl radical (˙OH), a radical oxygen species (ROS), in aliphatic and aromatic hydrocarbon biodegradation. after the biosynthesis of ˙OH by fungal enzymes via the quinone redox cycle, due to its extensive redox potential, ˙OH is deemed the most powerful oxidant in the fungal pathway [36, 37].

The application of microbial mixed cultures (MC) is an encouraging approach for the bioremediation of complex hydrocarbon, MC included many combinations, like bacterial (BMC), fungal (FMC), fungal and bacterial (FBMC), and sequential fungal–bacterial (SMC). The findings revealed that the SMC had the most potent of biodegradation (65.96%) in comparison to other mixed cultures [8]. Five fungal isolates were used to create the fungal consortium, as a fungal consortium supports a significant spectrum of ligninolytic enzymes, as well as a high ability to biodegrade diesel oil constituents and maintain appropriate conditions that lead to the transformation of oily substances into less toxic compounds [38]. Statistical experimental designs were used to optimize the process of diesel fuel biodegradation by the fungal consortium (*A*. *alternata* and *A*. *ustus*). Under optimized culture conditions, an overwhelming increase in biodegradation to 100% was observed. Thus, optimal conditions for the fungal consortium could be used in the treatment of diesel polluted soil [39].

### Effect of environmental factors on crude oil biodegradation

Based on the ANOVA test conducted, consortia number 11,12,13,14 and 15 have high significance towards enzyme activity efficiency against biodegradation of crude oil for this reason we selected these consortia to study the interaction between environmental factors and fungal consortia.

#### Crude oil concentration

The accumulation of contaminant hydrocarbons influences fungal biodegradation in the bioremediation process, and too high an accumulation contributes to a very decline in the performance of fungal biodegradation. As observed in Table 9, the crude oil concentration substantially affected the biodegradation of crude oil via the five-fungi consortia. The increase in the concentration of the crude oil indicates a decrease in the biodegradation by the all fungal consortia. The biodegradation efficiency of the fungi consortium no. 15 was still high compared to the other fungal consortia. The biodegradation efficiency of the three- and four-fungi consortia reached the greatest values of 63.97% and 61.87%, respectively, at the oil concentration of 5% (w/v). When the crude oil concentration was 20% (w/v), the biodegradation efficacy of every fungal consortium decreased significantly to less than 18%. 84 fungal isolates were tested to ability grow on crude oil, only 12 were ready to develop a crude oil with different concentrations with a range, 1% to 5%. Of the 12 isolates collected, 4 were classified as the most encouraging for oil bioremediation and these isolated belong to the Penicillium genus. 72 isolates were unable to develop at 1% and 5% crude oil, which can also explain the inability of some genus fungi to utilized crude oil as a carbon source at these concentrations. [40]. Two isolates Aspergillus oryzae and Mucor irregulars were could tolerate varying concentrations (5, 10, 15, and 20%) of used engine oil. biodegradation efficiency up to 39.40% and 45.85% at 20% engine oil for A. oryzae and M. irregulars. On the contrary, A. oryzae has a high level of hydrocarbon degradation by its great enzymes production. Seeming high level of enzyme production via fungi related to enhancing biodegradation of hydrocarbons faster than tolerance [2, 41].

**Table 9:** Effect of crude oil concentration on biodegradation efficiency of crude oil of 5 fungal consortia.

Consortium No.	Biodegradation efficiency (%)			
	Crude oil conc. 2.5%	Crude oil conc. 5%	Crude oil conc. 7.5%	Crude oil conc. 10%
11	55.93±1.66	25.97±1.63	18.50±0.75	10.57±1.36
12	55.23±1.75	29.37±0.95	20.63±1.89	12.17±1.48
13	53.97±1.56	26.60±1.90	21.97±1.40	12.60±1.01
14	61.87±2.34	28.03±2.89	21.60±2.82	13.97±1.72
15	63.97±0.95	32.53±2.57	27.77±1.72	17.70±0.80

#### Temperature

Temperature affects not only fungi behavior but also the chemical and physical characteristics of crude oil and the ability of fungi to biodegrade. We investigated the effect of a five-fungi consortia on biodegradation efficiency at 15–30°C. As shown in Table 10, the biodegradation ability of the five-fungi consortia increased with increasing temperature. In terms of biodegradation efficiency, during the temperature was 30°C, the maximum was achieved to 75.40% and 71.53% for the four- and three-fungi consortium, respectively. When the temperature was 15°C, the biodegradation efficiencies of all of fungal consortia ranged from 45.80% to 56.80%. The minimum biodegradation efficiency was greatly improved after using the fungal consortium no. 15, which increased by 18.6%, and can be used when a low temperature is not conducive to fungal activation and biodegradation. To search for temperature effects involved in the biodegradation of hydrocarbons, we had to correlate them with the enzymes involved in the degradation pathways. The main enzymes involved in the biodegradation of hydrocarbons are Cx, Lac, MnP, LiP, and LAP. These degradative enzymes require optimum temperature but their activity declines with very high and low temperatures [38]. Microorganisms, which biodegrade hydrocarbons, are remarkably effective at certain ranges of temperatures, which suitable for the enzyme-producing processes. Many microorganisms have an efficiency in the biodegradation of hydrocarbons at temperatures between 20°C and 35°C, which provides optimum biodegradation values. Owing to low temperatures, the enzyme activity was low and the viscosity of crude oil increases, the volatility of simple hydrocarbons decreases, and the solubility of these hydrocarbons increases. This makes the hydrocarbon reluctant to be biodegraded by microorganisms [42]. The optimum temperature for MnP was observed at 30° C, and MnP shows enhanced behavior at higher temperatures, which can be due to the strengthening of the structural rigidity of the protein molecule as it attaches to the strong support, decreasing the flexibility of the molecules [43].

**Table 10:** Effect of temperature on biodegradation efficiency of crude oil of 5 fungal consortia.

Consortium No.	Biodegradation efficiency (%)			
	15°C	20°C	25°C	30°C
11	45.80±1.70	56.37±0.81	61.07±1.61	67.13±1.63
12	47.10±2.62	56.03±1.60	63.93±2.16	66.83±2.22
13	46.10±1.74	55.13±1.26	63.53±2.17	67.63±1.50
14	50.30±2.59	58.83±1.78	67.33±3.20	71.53±1.10
15	56.80±2.33	64.70±2.36	74.13±2.60	75.40±2.17

#### Initial pH

As seen in Table 11, the biodegradation efficiency of all fungal consortia initially improved and decreased with an increased initial pH of the medium. While the initial pH was 7, the biodegradation efficiency was attained the best for all of the fungal consortia achieved the greatest values of 69.2% by fungal consortium no. 15. Fungal consortium no. 15 biodegradation efficiency was influenced by the initial pH values of 6 and 7, and the biodegradation efficiency variance amount reached up to 36.27%. However, when the initial pH 7 the biodegradation efficiency was up to 73.70%. The pH level for improved growth of the majority of bacteria is between pH 6.5 and 8.5, whereas the pH condition required for yeast and fungi is between pH 4.5 and 5.5. Thus, an optimal pH range for biodegradation of crude oil might be considered between pH 6.0 and 8.5. The pH can be highly variable and must be taken into consideration when improving biodegradation treatment methods. The environmental pH influences physiological processes such as transport through cell membrane and catalytic reaction balance well as enzyme activities [44]. The pH range for improved growth of most bacteria is between pH 6.5 and 8.5, in the pH 4.5–5.5 and in the pH 4.5–6.5 range for fungi. Therefore, an ideal pH range may be considered between pH 6.0 and 8.5 for the microbial biodegradation of crude oil [45]. MnP activity for *Aspergillus niger* consistently decreased in the range of pH 5.5–8.5, and was optimum at pH 5.5. MnP activity for *Penicillium freii* was lowest at pH 7.0 and optimum at pH 8.5 [46]. MnP activity for *Aspergillus terreus* was optimum at an alkaline pH of 12.5 and maintained its stability between the pH 11.0 and 12.5 [47]. The variation in the optimum pH of the enzyme activity between fungal isolates used in many of the cited studies could be due to the difference in substrates used or/and the strength of the isolate.

**Table 11:** Effect of initial pH on biodegradation efficiency of crude oil of 5 fungal consortia.

Consortium No.	Biodegradation efficiency (%)			
	pH 6	pH 7	pH 8	pH 9
11	27.10±2.10	61.97±1.02	54.57±2.15	22.90±2.59
12	25.53±2.73	62.77±2.29	57.63±2.46	20.97±2.54
13	27.33±1.91	63.13±2.66	56.10±2.11	25.33±2.32
14	32.67±2.08	70.40±3.12	63.07±2.42	26.63±2.65
15	37.43±3.13	73.70±4.31	66.23±2.24	25.60±2.36

#### Salinity

The experiments of crude oil biodegradation were conducted at salinity ranging from 2% to 8% to confirm the effectiveness of a mixture of three or four fungal isolates together as a consortium based on a synergistic effect that can tolerate wider salinity changes, and the findings are shown in Table 12. The effect of salinity on the biodegradation performance of crude oil was specifically influenced by fungal consortia. Initially, the biodegradation efficiency of all fungal consortia was increased and then declined with increasing salinity. the biodegradation efficiency of crude oil was very leading for all of the fungal consortia especially for the fungal consortium no. 15 (64.67%) at 4% of the salinity. When the salinity was 8%, the biodegradation efficiency of crude oil was very low for all of the fungal consortia, especially for the fungal consortium no. 11, which drop to the minimum value of 5.80%. The very significant variation in the biodegradation efficiencies of fungal consortium no. 15 was more than 60% when the salinity of the medium changed from 4% to 8%. Amending the salinity in soil plays an important role in the biodegradation of hydrocarbon-contaminated soil [48]. Possible reasons for the impact of salinity on the biodegradation cycle include the immediate inhibition of metabolic activity because of the high osmotic potential in the ecosystem, and altered solubility or sorption of toxic or essential ions [49]. Salinity has an adverse influence on the activity of some key complicated enzymes in the process of hydrocarbon biodegradation [50].

**Table 12:** Effect of salinity on biodegradation efficiency of crude oil of 5 fungal consortia.

Consortium No.	Biodegradation efficiency (%)			
	2%	4%	6%	8%
11	35.03±1.80	59.10±3.64	15.83±4.85	5.80 ±3.87
12	33.50±1.28	59.17±3.78	17.43±4.69	7.50±4.19
13	35.30±1.71	63.33±3.43	17.00±5.76	6.87±5.28
14	39.13±1.42	63.37±4.55	15.03±5.48	6.00±6.48
15	40.87±0.65	64.67±6.53	18.90±4.40	8.73±4.29

#### Degradation time

Table 13 presents the variation in the biodegradation efficiency of crude oil with time via five fungal consortia. The biodegradation efficiency of all of the fungal consortia improved initially and continued improving with time up until day 14. The biodegradation of crude oil by the fungal consortium no. 15 was evident and continued to improve strongly for 14 days, with a biodegradation efficiency of 75.00%. The biodegradation process of crude oil by fungal consortium no. 15 was powerful compared with that of the other fungal consortia. The significant variation in the biodegradation efficiencies of the fungal consortium no. 15 was more than 10% when the time of biodegradation changed from 11 to 14 days. The ligninolytic enzymes (LaC, LiP, and MnP) that produce white-rot fungi *Ganoderma lucidum* was used for the degradation of the PAH compounds (phenanthrene and pyrene). After 14 days, *Ganoderma lucidum* produced significant amounts (p < 0.0001) of ligninolytic enzymes and was able to biodegrade more than 90.00% of the PAHs [51]. White-rot fungi *Phanerochaete chrysosporium* was examined for its production of extracellular enzymes. MnP and LiP activity was measured during PAH biodegradation across 20 days. The maximum LiP and MnP activities were 1.92 ± 0.03 and 0.16 ± 0.005 U g^*-1*^ dry soil, respectively. The maximum value was achieved at day 11 with a biodegradation of more than 50.00% of PAHs [52].

**Table 13:** Effects of biodegradation time on crude oil degradation efficiency of 5 fungal consortia.

Consortium No.	Biodegradation efficiency (%)			
	5 Days	8 Days	11 Days	14 Days
11	34.10±1.08	44.30±1.50	54.57±2.51	66.03±2.55
12	31.60±1.08	43.17±2.70	52.47±2.47	65.07±2.08
13	34.90±0.82	42.77±3.05	58.80±2.95	68.70±1.65
14	36.17±1.30	57.70±18.66	60.27±1.76	70.83±1.55
15	41.90±1.18	53.63±3.74	64.33±2.64	75.00±3.02

### GC–MS analysis

#### Normal alkanes

Gas chromatograms of the blank and treated crude oil via fungal consortium no. 15 were shown in Fig 2a and 2b. Fig 1c shows the variation between blank of normal alkanes content and treatment samples. From this graph, we can see that fungal consortium no. 15 behaved differently in the biodegradation of normal alkanes. The biodegradation efficiency of normal alkanes by the fungal consortium no. 5 was in the range of 25%–84.7% with a mean of 67.1% (Fig 1d), and was the biodegradation efficiency of normal alkanes by fungal consortium no. 5 was divided into three groups. The first one had a very high rate of biodegradation of more than 70%, and included n-C12, n-C15, n-C16, and norpristane (NPr). The second had a high rate of biodegradation from 51% to 69%, and involved n-C18, iC-15, iC-16, n-C17 pristane phytane, and n-C13. The third group exhibited a medium rate of biodegradation of 50% and contained n-C14.

**Fig 2:** Normal alkanes gas chromatograms in crude oil samples before a) and after b) biodegradation by fungal consortium no. 15, c) changes of the major normal alkanes content in crude oil sample before and after biodegradation, d) biodegradation efficiency of the main normal alkanes.

#### PAHs

The gas chromatograms of PAHs of biodegradation by the fungal consortium no. 15 are shown in Fig 3a and 3b. As seen in Fig 1c, the content of 9 compounds of widespread PAHs is very low in the crude oil in treatment samples comparing to blank samples. The biodegradation efficiencies of PAHs of fungal consortium 5 in the range 44 to 72% with mean 67.1% Fig 1d the fungal consortium 5 showed positive biodegradation ability, with then biodegradation efficiencies above 50% for fluorene (F), methylfluorenes (MF), dimethylphenanthrenes (DMP), pyrene (Py), trimethylphenanthrene (TMP) and chrysene (C). Based on these observations of many researchers, it can be implied that using fungal consortia lead to a decrease in the hydrocarbons, in this case, the biodegradation is faster and easier for the decline hydrocarbons based on a complete system for enzymatic activities can be more efficient for the expansion of the range of biodegradable of crude oil [8, 38, 40].

**Fig 3:** PAHs gas chromatograms in crude oil samples before a) and after b) biodegradation by fungal consortium 15, c) changes of the major PAHs content in crude oil sample before and after biodegradation, d) biodegradation efficiency of the main PAHs.

## Conclusion

In this study, four oil-degrading fungal isolates (AA-1, AF-3, AT- and TH-5) were isolated from the date palm soil in Saudi Arabia. They were identified to *Alternaria alternata*, *Aspergillus flavus*, *Aspergillus terreus*, and *Trichoderma harzianum*, respectively. The mixed four fungal isolates showed the most powerful biodegradation efficiency of crude oil of 73.6%. Fungal consortium no. 15 included all four fungi (1:1:1:1) achieved better than another consortium in variations of environmental factors containing incubated temperature, initial pH and salinity of the medium. To get high performance of the biodegradation efficiency after 14 days for biodegradation, the concentration of crude oil (5%, w/v), with a temperature of 25°C, initial pH of 7.0, the salinity of 25% and treatment with of fungal consortium no. 5. The average of biodegradation efficiency by the fungal consortium no. 15 of normal alkanes (67.1%) was clear high than that of PAHs (56.8%).

## Supporting information

S1 Fig (a) Normal probability plot for residual value, (b) residual plots against fitted value, (c) histogram of residual value, (d) residual plot against observation order of individual fungi and fungal consortium producing laccase. (DOCX)

S2 Fig (a) Normal probability plot for residual value, (b) residual plots against fitted value, (c) histogram of residual value, (d) residual plot against observation order of individual fungi and fungal consortium producing lignin peroxidase. (DOCX)

S3 Fig (a) Normal probability plot for residual value, (b) residual plots against fitted value, (c) histogram of residual value, (d) residual plot against observation order of individual fungi and fungal consortium producing lipase. (DOCX)

S4 Fig (a) Normal probability plot for residual value, (b) residual plots against fitted value, (c) histogram of residual value, (d) residual plot against observation order of individual fungi and fungal consortium producing manganese peroxidase. (DOCX)
